The article "CircANXA2 Promotes Myocardial Apoptosis in Myocardial Ischemia-Reperfusion Injury via Inhibiting miRNA-133 Expression" was retracted in 2024. Reasons: signs of a paper mill; suspected computer-generated content; unreliable results or conclusions; concerns about the data.

# CircANXA2 Promotes Myocardial Apoptosis in Myocardial Ischemia-Reperfusion Injury via Inhibiting miRNA-133 Expression

**DOI:** 10.1155/2020/8590861

**Published:** 2020-06-24

**Authors:** Liang Zong, Weixin Wang

**Affiliations:** Department of Cardiac Surgery, Affiliated Hospital of Jining Medical University, Jining, Shandong, China

## Abstract

**Objective:**

This project is aimed at investigating whether CircANXA2 can promote the apoptosis of myocardial cells by inhibiting miR-133 expression and thereby participate in the development of myocardial ischemia-reperfusion injury. *Materials and Method*. Quantitative real-time polymerase chain reaction (qRT-PCR) was used to detect the expression level of CircANXA2 in H9c2 cells after hypoxia/reoxygenation (H/R) treatment. Evaluation of myocardial injury markers in H9c2 cells was performed using commercial kits, including lactate dehydrogenase (LDH), malonaldehyde (MDA), superoxide dismutase (SOD), and glutathione peroxidation (GSH-PX). MTT analysis and flow cytometry were used to detect myocardial cell proliferation and apoptosis, respectively. Western blot was used to detect the protein expression of apoptosis-related genes.

**Result:**

qRT-PCR results showed that compared with the control, the expression of CircANXA2 was upregulated and the expression level of miR-133 was significantly decreased in H/R-treated H9c2 cells. CircANXA2 overexpression increased LDH, MDA, SOD, and GSH-PX activity in H/R-treated H9c2 cells. At the same time, CircANXA2 overexpression inhibited the proliferation of H/R-treated cells, and CircANXA2 was able to induce cardiomyocyte apoptosis. Western blot results showed that after overexpression of CircANXA2, the proapoptotic genes Bax and cytochrome C was upregulated, while the antiapoptotic gene Bcl-2 was downregulated. In H9c2 cells, upregulating miR-133 can reverse the inhibition of proliferation induced by CircANXA2 overexpression and increase apoptosis.

**Conclusions:**

CircANXA2 promotes cardiomyocyte apoptosis in myocardial ischemia-reperfusion injury by inhibiting the expression of miR-133. CircANXA2 may be a potential target for myocardial ischemia-reperfusion injury.

## 1. Introduction

Ischemic heart disease is one of the common diseases of the cardiovascular system in clinical practice [1–4]. Reperfusion of human ischemic coronary artery can effectively reduce the total mortality. However, the restoration of blood flow to previously ischemic cells will aggravate the symptoms of reperfusion injury, including myocardial cell dysfunction and cell death. Myocardial ischemia-reperfusion injury (MIRI) refers to the myocardial blood supply interruption within a short period of time; after the recovery of blood supply within a certain period of time, the primary ischemic myocardial injury is more serious than that during ischemia. MIRI mechanism has not been fully elucidated; it is generally believed that the reperfusion outbreak of free radicals, calcium overload, mitochondrial damage, adenosine triphosphate (ATP) energy metabolic disorders, cell autophagy, apoptosis and necrosis, and inflammation is ischemia-reperfusion injury (IRI) pathological process; the main reasons for the occurrence and development connect with each other between the injury mechanisms, often triggering or indirectly causing damage to another [5–7].

circRNA is a type of closed circular noncoding RNA that does not contain a 5′ end cap and a 3′ end Poly (A) tail and is covalently bound by the head and tail [8–10]. According to its source in the genome and its constituent sequences, it is divided into exon circRNA (ecircRNA), intron circRNA (ciRNA), and exon-intron circRNA (EIciRNA). circRNA plays an important role in the pathogenesis of coronary heart disease, and it is also of great significance in predicting the occurrence, development, and prognosis of coronary heart disease. At present, there are few studies on circRNA and coronary heart disease, and the specific mechanism involved in coronary heart disease is not clear, and further research is needed. Li et al. found that the expression of hsa_circ_0003575 was significantly upregulated in the human umbilical vein endothelial cell injury model induced by oxidized low-density lipoprotein. Silencing this gene can lead to the proliferation of endothelial cells and the formation of blood vessels. Researchers believe that hsa_circ_0003575 can regulate endothelial cells during atherosclerosis [11].

MicroRNAs (miRNAs) are endogenous noncoding short RNA molecules that regulate gene expression by inhibiting translation or cleaving RNA in a specific sequential manner (complementarily paired with the target mRNA). miRNA-133 is involved in the occurrence and development of various cardiovascular diseases, especially myocardial remodeling and arrhythmia. At present, the mechanism of action of miRNA-133 is not fully understood [12].

This study reveals the role of miR-133 in myocardial ischemia-reperfusion injury. To our knowledge, no studies have been conducted to explore the role of CircANXA2 in the regulation of myocardial cell apoptosis. The purpose of this study was to elucidate the role of CircANXA2 in myocardial ischemia-reperfusion injury and to investigate its mechanism affecting myocardial ischemia-reperfusion injury.

## 2. Materials and Method

### 2.1. Cell Culture and H/R Treatment

Rat embryonic cardiomyocyte H9c2 was purchased from ATCC (American Type Culture Collection, Manassas, VA, USA). H9c2 cells were cultured in Dulbecco's modified Eagle medium (DMEM; containing 10% fetal bovine serum (fetal bovine serum; Gibco, Rockville, Maryland, USA)).

### 2.2. Construction of Myocardial Ischemia-Reperfusion Injury Cell Model (H/R Cells)

H9c2 cells were cultured in serum-free DMEM and maintained for 4 hours in an anaerobic incubator with 5% CO_2_ and 95% N_2_. Subsequently, H9c2 cells were cultured in DMEM containing 10% glycerol for 3 hours (5% carbon dioxide and 95% air) and finally reoxygenated for 24 h. Cells were then collected for subsequent experiments.

### 2.3. Cell Transfection

Well-grown cardiomyocytes were seeded in 6-well plates in serum-free medium. According to the operating requirements of Lipofectamine 2000 (Invitrogen, Carlsbad, CA, USA), transfection was performed when the fusion reached 60%. First, Lipofectamine 2000 and plasmid were diluted in serum-free medium and mixed for 20 minutes at room temperature. The mixture was then added to each cell culture well and incubated. After 4-6 hours of culture, the medium was changed. The transfection plasmid used in this study was constructed by GenePharma Co., Ltd. (Shanghai, China). siRNAs were also transfected with Lipofectamine 2000. Refer to the transfection reagent instructions for the transfection procedure.

### 2.4. qRT-PCR

According to instructions of PrimeScript RT reagent kit (TaKaRa, Otsu, Shiga, Japan), the total RNA of cells after different treatments was extracted by TRIzol method (Invitrogen, Carlsbad, CA, USA). After that, reverse transcription was performed. RNA concentration was measured by using a spectrometer. qRT-PCR was performed according to the instructions of SYBR Premix Ex Taq™ (TaKaRa, Otsu, Shiga, Japan). Relative gene expression was calculated using the 2-*Δ*Ct method.

### 2.5. Detection of LDH, MDA, SOD, and GSH-PX

Cells were collected after different treatments, and the activities of LDH, MDA, SOD, and GSH-PX were measured according to the instructions of the commercial kit.

### 2.6. CCK-8

Transfected cells were passaged into 96-well plates in a cell density of 2 × 10^3^/*μ*L. Pipette 10 *μ*L of CCK-8 (Dojindo, Kumamoto, Japan) solution into each cell culture well, and continue the culture. After 72 hours, the absorbance of each sample at 450 nm was measured using a microplate reader (Bio-Rad, Hercules, CA, USA).

### 2.7. Western Blot

RIPA lysis buffer was used to lyse myocardial cells after different treatments under protease inhibitor (Sigma-Aldrich, St. Louis, Missouri, USA) conditions. Cell proteins were collected, and the protein concentration of each cell lysate was quantified using a BCA (bicinchoninic acid) protein detection kit (Pierce, Rockford, IL, USA). 50 *μ*g protein samples were added to a 10% SDS-PAGE (sodium dodecyl sulfate-polyacrylamide gel electrophoresis) to gel loading well. After the protein is separated by gel electrophoresis, the protein is transferred to a PVDF (polyvinylidene fluoride) membrane (Millipore, Billerica, MA, USA). Nonspecific binding antigen was blocked with 5% skim milk and then incubated with primary antibody: Bax (Abcam, 1 : 1000), Bcl-2 (Abcam, 1 : 1000), cleaved caspase-3 (Abcam, 1 : 1000), and cleaved caspase-9 (Abcam, 1 : 1000) at 4°C overnight, and then incubated with horseradish peroxidase-conjugated secondary antibody at room temperature (1 hour). Finally, images of protein bands were captured using the Tanon detection system using enhanced chemiluminescence (ECL) reagents (Thermo, Waltham, MA, USA).

### 2.8. Apoptosis Detection

For TUNEL experiments, TUNEL apoptosis detection kit (Yisheng, Shanghai, China) was used to detect apoptosis. The detection procedure was performed according to the kit instructions. Flow cytometry is also used to detect the apoptotic rate. The operation steps are performed according to the instructions of the apoptotic staining kit.

### 2.9. Reporter Gene Construction and Luciferase Assay

A cDNA fragment containing the CircANXA2 binding site was amplified by PCR. The amplified product was cloned into a PGL3 vector (Promega, Madison, WI, USA), which was located downstream of the stop codon of the luciferase gene. A miR-133 mutant was constructed. For luciferase detection in HEK-293T, luciferase activity was detected using the dual luciferase reporter kit (Promega) according to the manufacturer's instructions.

### 2.10. Pull-Down Experiment with Biotinylated miR-133 Probe

A DNA probe synthesizes biotinylated miR-133 interacting binding moiety. The probes were incubated with streptavidin-coated agarose beads at 25°C for 2 hours to generate probe-coated agarose beads. The H9c2 cell lysate was incubated with the probe-coated microspheres. After washing with the washing/binding buffer, the RNA complex bound to the microspheres was eluted and extracted. Using purified RNA as a template, CircANXA2 was analyzed by qRT-PCR.

### 2.11. Statistical Analysis

Statistical Product and Service Solutions (SPSS) 19.0 statistical software was used for data analysis. Data is expressed as mean ± standard deviation (*x* ± *s*). Comparisons between two groups were tested by *t* test, and comparisons between multiple groups were analyzed by ANOVA. *p* < 0.05 was considered statistically significant.

## 3. Results

### 3.1. CircANXA2 Expression Is Upregulated in H/R Cells

To understand the role of CircANXA2 in the heart, we detected its expression level under oxidative stress. A time-dependent increase in CircANXA2 level was observed in H9c2 cells upon treatment with 100 *μ*M H_2_O_2_ (Figure 1(a)). The experiment was divided into control group (conventionally treated H9c2 cells) and H/R-treated H9c2 cell line (H/R cells). Hypoxia/reoxygenation (H/R) treatment also increased the CircANXA2 level in H9c2 cells (Figure 1(b)). Experimental results show that CircANXA2 is upregulated in myocardial ischemia.

### 3.2. Overexpression of CircANXA2 Promotes Expression of Markers of Myocardial Ischemia-Reperfusion Injury

To further investigate the function of CircANXA2, we measured levels of cardiac injury markers that overexpressed CircANXA2 in H/R-treated cells. The results showed that the overexpression plasmid could effectively upregulate the expression of CircANXA2 (Figure 2(a)). Meanwhile, the overexpression of CircANXA2 increased the activity of LDH, MDA, SOD, and GSH-PX (Figures 2(b)–2(e)).

### 3.3. Overexpression of CircANXA2 Promotes Apoptosis of Cardiomyocytes

We further investigated the regulation of CircANXA2 on H/R cell proliferation. CCK-8 analysis showed that the cell proliferation was weakened after overexpression of CircANXA2 (Figure 3(a)). Flow cytometry indicated that overexpression of CircANXA2 promoted apoptosis of H9c2 cells (Figure 3(b)). To further explore the mechanism of CircANXA2 in regulating cell apoptosis, the expression levels of proapoptotic genes Bax and cytochrome C and antiapoptotic gene Bcl-2 were detected. qRT-PCR data showed that after overexpression of CircANXA2, the mRNA levels of Bax and cytochrome C increased, while the expression of Bcl-2 decreased (Figures 3(c)–3(e)). Western blotting showed that cleaved caspase-3 and cleaved caspase-9 proteins increased with the overexpression of CircANXA2. The results showed that the overexpression of CircANXA2 promoted the apoptosis of cardiomyocytes (Figures 3(f) and 3(g)).

### 3.4. CircANXA2 Binds Directly to miRNA-133 in Cardiomyocytes

In order to study the target genes bound by CircANXA2, we predicted through StarBase that CircANXA2 could directly bind to miR-133 (Figure 4(a)). Further dual luciferase reporter assay results confirmed the binding of CircANXA2 to miR-133 (Figure 4(b)). RNA pull-down (miRNA-133 probe) experiments also showed that CircANXA2 was able to bind to miR-133 (Figure 4(c)). Biotin-miRNA-133 probe be bound to the CircANXA2 enrichment landing significantly. Further testing the effect of CircANXA2 on the expression of miR-133 showed that CircANXA2 can inhibit the expression level of miRNA-133, and knockdown of CircANXA2 can increase the expression level of miR-133 (Figures 4(d) and 4(e)). The expression of miRNA-133 in cardiomyocytes showed that miR-133 was downregulated during myocardial ischemia (Figure 4(f)).

### 3.5. Overexpression of miRNA-133 Reverses the Apoptosis Promotion Effect of CircANXA2

Cell proliferation experiments show that miR-133 can reverse the effect of CircANXA2 on inhibiting cell proliferation. Compared with the control group, CircANXA2 treatment inhibited myocardial cell proliferation, and overexpression of miR-133 reversed the inhibitory effect of CircANXA2 (Figure 5(a)). Apoptosis test results showed that CircANXA2 can induce cardiomyocyte apoptosis, and overexpression of miR-133 reversed the proapoptotic effect of CircANXA2 (Figure 5(b)). The results of TUNEL staining were consistent with the results of flow cytometry (Figures 5(c) and 5(d)). Bax protein expression test results showed that CircANXA2 can induce upregulation of Bax protein expression in cardiomyocytes, while overexpression of miR-133 reversed the effect of CircANXA2 on promoting Bax expression. The results of Bcl-2 protein expression were opposite to those of Bax. CircANXA2 could inhibit Bcl-2 expression, while overexpression of miR-133 reversed the effect of CircANXA2 (Figures 5(d)–5(g)).

## 4. Discussion

Coronary heart disease is one of the leading causes of death and disability worldwide [13]. The main treatment methods are drugs, percutaneous coronary intervention, and coronary artery bypass grafting. Various revascularization methods can alleviate myocardial injury and necrosis caused by ischemia by restoring myocardial perfusion in time and effectively. However, restoration of blood reperfusion after myocardial ischemia can itself further lead to myocardial cell damage and even necrosis, a phenomenon known as myocardial ischemia-reperfusion injury [14–18]. However, up to now, there is still no effective clinical treatment method to avoid myocardial ischemia-reperfusion injury, which seriously restricts the therapeutic effect of coronary heart disease. Therefore, it is of great significance to study its pathophysiological mechanism and find effective prevention and treatment measures to improve the prognosis of patients with coronary heart disease.

Circular RNA (circRNA) is a noncoding RNA that has the function of targeted regulation of small RNA (miRNA) or messenger RNA (mRNA) [19]. It is involved in atherosclerosis, immune response, angiogenesis, apoptosis, cell proliferation, and various mechanisms of coronary heart disease (CHD), including cell senescence and cell autophagy. The circRNA/miRNA/mRNA interactive network based on circRNA helps to reflect the occurrence and development of CHD systematically and dynamically [20, 21]. At the same time, circRNA provides new targets and new strategies for the targeted and precise treatment of CHD in the future through pharmacological intervention or artificial overexpression/knockdown of the abnormal expression of circRNA and editing of the circRNA sequence. Myocardial cell abnormal apoptosis is an important factor in the development of CHD. Studies have shown that myocardial ischemia and hypoxia can induce changes in the circRNA expression profile of mouse heart tissue, and the expression of CiRS-7 is upregulated [22]. Another study showed that miR-652-3p can directly downregulate mitochondrial protein (MTP) 18 expression, inhibit mitochondrial division and myocardial cell apoptosis, and improve myocardial infarction. circRNA-MFACR downregulates the expression of miR-652-3p, preventing the myocardial protection of miR-652-3p, and this effect can be reversed by the low expression of circRNA-MFACR. Therefore, by targeting the regulation of miR-652-3p/MTP18, circRNA-MFACR can promote the apoptosis of myocardial cells and accelerate the progress of myocardial infarction [23]. In addition, reactive oxygen species (ROS) can induce CircANXA2 overexpression, while CircANXA2 can promote the apoptosis of myocardial cells. Its potential mechanism of action is to competitively bind miR-133a-3p, thereby increasing the expression of proapoptotic factor cell death-inducing protein. During knockdown of CircANXA2 in cardiomyocytes and cardiac tissues of mice, CDIP1 expression was reduced, apoptosis was suppressed, and myocardial ischemia/reperfusion (I/R) injury was improved [24]. It can be seen that CircANXA2 is a promoter of myocardial ischemia, mediates the downstream miR-133a-3p/CDIP1 regulatory pathway, and participates in the apoptosis process of myocardial I/R injury.

In this study, CircANXA2 was found to be highly expressed in H/R-treated cells compared with the control group. Overexpression of CircANXA2 can improve the activity of LDH, MDA, SOD, and GSH-PX in H/R cells. In vitro experiments showed that overexpression of CircANXA2 reduced cell proliferation and induced apoptosis. The overexpression of CircANXA2 also upregulated Bax and cytochrome C, while downregulating Bcl-2. In H/R-treated cells, the expression of miR-133 was downregulated, and CircANXA2 negatively regulated the expression of miR-133. We found that the overexpression of miR-133 reversed the effect of CircANXA2.

miRNAs is a general term for a large class of small molecule noncoding single-stranded RNAs that are highly conserved during evolution of about 22 single nucleotides in length. The mature miRNA is base-paired with the 3′ noncoding region (3′-UTR) of the target gene mRNA, and the expression of the target gene is downregulated by cleaving the mRNA or inhibiting translation. miRNAs have been shown to be involved in the pathogenesis of a variety of cardiovascular diseases including atherosclerosis, coronary artery disease, myocardial infarction, heart failure, and arrhythmia. The expression of miRNA has strict tissue-cell specificity and time-specific developmental stage. Some research found that 220 kinds of human miRNA are expressed in cardiac tissues; miRNA-133, which is specifically expressed in the heart, plays an important regulatory role in cardiac development, myocardial apoptosis, and myocardial remodeling [25, 26]. miR-133 has an antiapoptotic effect. Xu et al. [27] confirmed that miR-133 inhibited the apoptosis of cardiac myocytes by inhibiting the expression of the apoptotic protein caspase-9. Chen et al. [28] confirmed that miR-133 can directly regulate the expression of collagen *α* 1 (I) chain; it is suggested that there is a direct connection in miR-133 with cardiac myofibrinolysis.

In summary, we have observed that CircANXA2 promotes myocardial apoptosis during myocardial ischemia-reperfusion by inhibiting the expression of miR-133 and aggravates myocardial ischemia-reperfusion injury. This study provides a potential therapeutic target for myocardial ischemia-reperfusion injury and expands the understanding of the role of circular RNA in myocardial ischemia-reperfusion injury.

## Figures and Tables

**Figure 1:** CircANXA2 is upregulated in H/R cells. (a) H9c2 cells were treated with 100 *μΜ* H_2_O_2_. Total RNA was isolated and reverse-transcribed. The CircANXA2 level was analyzed by qRT-PCR. ∗*p* < 0.05 versus 0 h (*N* = 3). (b) Detection of CircANXA2 expression in H/R cells. Grouping: control group (conventionally treated H9c2 cells); H/R-treated H9c2 cell line (H/R cells).

**Figure 2:** Overexpression of CircANXA2 promotes expression of markers of myocardial ischemia-reperfusion injury. (a) CircANXA2 expression detection. (b) Detection of LDH expression. (c) Detection of MDA expression. (d) Detection of SOD expression. (e) Detection of GSH-PX expression.

**Figure 3:** Overexpression of CircANXA2 promotes cardiomyocyte apoptosis. (a) Cell proliferation ability test. CCK-8 assay showed that cell proliferation was attenuated after overexpression of CircANXA2. (b) Flow cytometry to detect apoptosis. Flow cytometry suggested that overexpression of CircANXA2 promoted apoptosis of H9c2 cells. (c) Detection of Bax protein expression. (d) Detection of Bcl-2 protein expression. (e) Cytochrome C expression level detection. (f) The protein expression levels of 3 and 9 were detected by Western blot. (g) Detection of cleaved caspase-3 expression. (h) Detection of cleaved caspase-9 expression.

**Figure 4:** CircANXA2 binds directly to miRNA-133 in cardiomyocytes. (a) CircANXA2 targets miRNA-133 binding site information. (b) The binding of CircANXA2 to miR-133 was verified by the dual luciferase report assay. (c) RNA pulled down (miRNA-133 probe). (e) Detection of miRNA-133 expression level. (f) miRNA-133 expression in cardiomyocytes.

**Figure 5:** Overexpression of miRNA-133 reverses the apoptosis promotion effect of CircANXA2. (a) Cell proliferation experiments after different treatments. (b) Apoptosis results after different treatments. (c, d) TUNEL staining intensity of cells after different treatments. (e–g) Detection of Bax and Bcl-2 protein expression.

## Data Availability

All the raw data could be accessed by contacting the corresponding author if any qualified researcher need.
